The article "Designing biomaterials for the delivery of RNA therapeutics to stimulate bone healing" was published in 2021. Journal: Mater Today Bio.

# Designing biomaterials for the delivery of RNA therapeutics to stimulate bone healing

**DOI:** 10.1016/j.mtbio.2021.100105

**Published:** 2021-03-06

**Authors:** L. Andrée, F. Yang, R. Brock, S.C.G. Leeuwenburgh

**Affiliations:** a Department of Dentistry – Regenerative Biomaterials, Radboud Institute for Molecular Life Sciences, Radboudumc, Philips van Leydenlaan 25, Nijmegen, 6525 EX, the Netherlands; b Department of Biochemistry, Radboud Institute for Molecular Life Sciences, Radboudumc, Geert Grooteplein 28, Nijmegen, 6525 GA, the Netherlands

**Keywords:** Oligonucleotide delivery, RNA delivery, mRNA, Controlled release, Bone regeneration

## Abstract

Ribonucleic acids (small interfering RNA, microRNA, and messenger RNA) have been emerging as a promising new class of therapeutics for bone regeneration. So far, however, research has mostly focused on stability and complexation of these oligonucleotides for systemic delivery. By comparison, delivery of RNA nanocomplexes from biomaterial carriers can facilitate a spatiotemporally controlled local delivery of osteogenic oligonucleotides. This review provides an overview of the state-of-the-art in the design of biomaterials which allow for temporal and spatial control over RNA delivery. We correlate this concept of spatiotemporally controlled RNA delivery to the most relevant events that govern bone regeneration to evaluate to which extent tuning of release kinetics is required. In addition, inspired by the physiological principles of bone regeneration, potential new RNA targets are presented. Finally, considerations for clinical translation and upscaled production are summarized to stimulate the design of clinically relevant RNA-releasing biomaterials.

## 1 Introduction

Human bone has a strong regenerative capacity that allows restoration of its function and structure after damage [1]. However, bone grafts or bone substitute materials are required to support the regeneration of bone tissue when this regenerative capacity is compromised by, for example, degenerative bone diseases or formation of bone defects that exceed a certain critical size. Compared to native bone grafts, which contain a plethora of osteogenic factors, the regenerative capacity of man-made bone substitute materials, such as metal implants, calcium phosphate bioceramics, or polymeric fillers, is very limited [2,3]. Therefore, extensive research has been dedicated to biological functionalization of these biomaterials with osteogenic factors to boost their regenerative capacity. To this end, a wide variety of bioactive molecules has been considered as candidate therapeutics, including hormones (e.g., parathyroid hormone, steroids, estrogen), statins, or anti-osteoclastic drugs (e.g., bisphosphonates) [4,5]. Generally, osteogenic growth factors such as bone morphogenetic proteins (BMPs) are recognized as the most potent biomolecules to support bone regeneration using biomolecule-loaded biomaterials.

The article "Designing biomaterials for the delivery of RNA therapeutics to stimulate bone healing" was published in 2021. Journal: Mater Today Bio.

In 1965, Marshall R. Urist demonstrated that demineralized bone matrix could stimulate bone growth in ectopic sites [6], leading to the discovery of BMPs ​[7]. Ever since, these proteins have been studied extensively for application in bone regeneration. In 2002, the first BMP-2-delivering device for bone regeneration was commercially marketed [8]. However, high supraphysiological amounts of growth factor were required to achieve bone regeneration due to rapid and uncontrolled delivery, release into systemic circulation, as well as premature degradation of the loaded protein [9,10]. The high concentration of BMP-2 used in these devices induced severe (systemic) side effects, including osteolysis, dysphagia, and damage of nerve tissue (neurologic events, retrograde ejaculation, leg pain, functional loss) [[11], [12], [13]]. These severe side effects were observed for both on-label and off-label use in, for example, cervical surgery [14]. This negative outcome of the first BMP-2 delivering device has complicated the commercialization and Food and Drug Administration (FDA) approval of future growth factor-containing medical devices. Moreover, industrial production of these factors at clinical grade is very costly.

### 1.1 Emergence of gene therapy and RNA therapeutics

To avoid loss of bioactivity, safety issues and excessive production costs associated with the large amounts of proteinaceous growth factors that are required because of rapid degradation (Table 1), gene therapy has emerged as an alternative strategy, with first clinical trials taking place in the early 1990s [15]. Instead of delivering proteins, cells are transfected with DNA to induce endogenous expression of growth factors [16]. Compared to protein delivery, gene therapy is effective for long time periods without the need of repetitive administration [17]. However, DNA requires a properly chosen promotor region to control gene expression; otherwise, there is a risk of overexpression. Also, DNA has to enter the nucleus and, ​for this reason, transfection of non-dividing cells still poses a challenge. Moreover, viral vectors are still preferred over synthetic delivery systems due to their much higher transfection efficiency ​but may be immunogenic. For DNA delivery in general, random genome insertion and carcinogenicity are safety concerns [15,17,18]. Nevertheless, several (cell-based) gene therapies are approved by the FDA for clinical use [19]. As a safe and transient alternative, RNA therapies including small interfering RNA (siRNA), microRNA (miRNA) and messenger RNA (mRNA) have recently gained considerable interest. In contrast to DNA, RNA exerts its function in the cytosol, eliminating the need for nuclear uptake and omitting the risk of random insertion into the genome (Table 1). While DNA delivery still depends on viral vectors for efficient cellular transfection, non-viral vectors are commonly used for RNA delivery and show good transfection efficiency [17,18,20].

The article "Designing biomaterials for the delivery of RNA therapeutics to stimulate bone healing" was published in 2021. Journal: Mater Today Bio.

**Table 1:** Comparison of protein-, gene- and oligonucleotide-therapy^a^.

	Growth factor therapy	Gene therapy	RNA therapy
Mode of action	Binding to receptor to elicit signaling pathway	Endogenous transcription and translation into target protein	Modulation of endogenous protein expression
Location of action	Plasma membrane	Nucleus	Cytosol
Delivery vector	None	Viral or non-viral methods	Non-viral methods
Effect onset and duration	Fast and transient	Slow and long-term	Fast and transient, controllable kinetics
Transfection	Dividing and non-dividing cells	Dividing cells, difficult in nondividing cells	Dividing and non-dividing cells
Advantages	No vectors needed, well studied	Long-lasting effect, endogenous protein expression, not limited to growth factor expression (e.g., receptors)	Transient effect, endogenous protein expression, not limited to growth factor expression (e.g., receptors), good control of dose
Disadvantages	Fast degradation, loss of bioactivity, high production costs, risk of overstimulation	Risk of random genomic integration and carcinogenesis, nonviral vectors show low efficacy, risk of unwanted immune response	Fast degradation and low transfection efficacy without complexation, risk of unwanted immune response

a Based on [15,17,18,20,21].

Once in the cytosol, RNAs act by forming complexes with endogenous proteins [21]. siRNA and miRNA both associate with the RNA-induced silencing complex (RISC) to target and degrade mRNA (Fig. 1), leading to a reduced protein expression [22,23]. miRNA is single-stranded, whereas siRNA is double-stranded. Furthermore, miRNAs are also encoded in the genome and act as post-transcriptional regulators of gene expression by targeting the 3′ untranslated region (UTR) of mRNAs [22,24,25]. In contrast, siRNA is a double-stranded, mainly exogenous RNA originally coming from viruses and transposons that targets mRNAs and triggers their degradation [22,23]. While one miRNA can bind to various mRNAs, naturally occurring siRNA requires full complementarity for binding its target [24,25]. However, therapeutic siRNAs are man-made and can be designed to target any sequence, including the 3′UTR to mimic the effect of natural miRNAs.

The article "Designing biomaterials for the delivery of RNA therapeutics to stimulate bone healing" was published in 2021. Journal: Mater Today Bio.

**Fig. 1:** **RNA mechanisms of action**. Left: A gene is transcribed into mRNA. After export through the nuclear pores into the cytosol, the mRNA is translated into the corresponding protein by the ribosome. In particular along the secretory route, the protein will undergo posttranslational modifications. Right: Single-stranded miRNA is transcribed in the nucleus and gets exported into the cytosol where it associates with the RNA-induced silencing complex (RISC). In contrast, siRNA is a double-stranded RNA of exogenous origin, which gets processed into a single-strand molecule in the cytosol before association with RISC. The miRNA or siRNA strand guide the RISC complex to the target mRNA by (partial) sequence complementarity. miRNA either leads to degradation of the target mRNA or inhibits its translation, whereas siRNA usually leads to the degradation of the target mRNA.

mRNA associates with ribosomes to induce translation, leading to protein production [21] (Fig. 1). Compared to *in vitro* synthesis of recombinant proteins in heterologous expression systems, the mRNA-based approach assures correct post-translational modification of proteins, which are often highly challenging to recapitulate during *in vitro* synthesis [20]. Moreover, mRNA is not restricted to expression of growth factors but also enables the expression of proteins that act inside the cell or as transmembrane cell surface receptors, thereby widening the scope of therapeutic targets. The effects of RNAs are only transient, which allows ​for temporal control over gene silencing and protein expression, eliminating the need for supraphysiological doses and thus reducing the risk of growth factor overdosing [17,26]. Yet, for mRNA, expression can be extended over several days, which is superior to the short biological half-life of recombinant proteins.

Until now, several siRNA-based therapies have entered clinical trials, and one has been clinically approved, but applications are still very much limited to hepatic pathologies and cancer [26]. Similarly, clinical trials on mRNA-based therapies have mostly been focusing on cancer immunotherapy and prophylactic vaccines [27,28]. However, protein replacement therapy is also being tested. Prominent examples of trials on protein replacement therapy are expression of cystic fibrosis transmembrane regulator protein in cystic fibrosis [29,30] and vascular endothelial growth factor A (VEGF-A) [31]. The latter has been tested in phase I clinical trial for the treatment of ulcers associated with type II diabetes (NCT02935712) and is currently in phase II clinical trial for the treatment of heart failure (NCT03370887). Moreover, mRNA delivery also shows potential for gene editing [32], expression of engineered antibodies [33], and cellular reprogramming [34], which may offer new opportunities for advanced tissue engineering. The transient expression of VEGF to reduce tissue damage after myocardial infarction is a notable example showing the strong potential of local mRNA delivery to stimulate expression of a growth factor [35]. The full breadth of the potential of mRNA therapeutics for diverse applications has been reviewed elsewhere [36,37].

The article "Designing biomaterials for the delivery of RNA therapeutics to stimulate bone healing" was published in 2021. Journal: Mater Today Bio.

### 1.2 Challenges of RNA therapeutics

Although RNA-based strategies, and in particular mRNA-based strategies, offer new tools for tissue engineering, several hurdles regarding transfection efficacy, RNA stability, and immunogenicity need to be overcome. RNAs are negatively charged molecules, which compromises ​direct diffusion through the lipid bilayer of cell membranes [20,24]. Therefore, current RNA-based therapies use complexation agents based on cationic molecules to condense the RNA into nanocomplexes by electrostatic interactions, thereby facilitating cell transfection. Complexation agents can be broadly categorized into five groups: lipids, polypeptides, polymers, dendrimers and hybrids thereof. These categories have been extensively reviewed elsewhere [15,18,20,21,37]. In addition, direct conjugation with cholesterol, vitamin E or N-acetylgalactosamine (GalNAc) has been tested, but this approach is still limited to smaller RNAs (siRNA and miRNA) [21,36].

RNA complexation does not only further cellular internalization and endosomal escape ​but also protects the RNA from degradation by ribonucleases [18,26]. Nevertheless, RNA stability and translation efficiency remain a challenge. mRNA, for example, has a median intracellular half-life time of 7 ​h [20]. To improve stability and activity, researchers often chemically modify one or more of the structural elements of RNA. The 5′ cap plays an important role in the initiation of translation and interacts with a complex that regulates RNA decay. The selection of appropriate cap structures and synthetic cap mimetics have been shown to increase translation efficiency. In addition, translation speed can be increased through codon optimization within the coding sequence. By selecting codons of the most frequently occurring transporter RNAs for each amino acid, the peptide chain can be assembled faster. Selection of 5′ and 3′ UTRs from mRNAs with long half-life times (e.g., 5′ UTR of human heat shock protein 70 mRNA, 3’ UTR of α- or β-globin mRNA) help stabilizing the mRNA. Similarly, the length of the poly(A)-tail affects mRNA stability through protection against degradation by nucleases ​and regulates translation efficiency. A length of 120–150 nucleotides has been reported necessary for optimal inhibition of mRNA degradation [17,20,38].

mRNA brought into a cell from the outside is a sign of viral infection and activates the immune system. To alleviate the immunogenic effects of mRNA therapeutics, chemically modified ribose sugars and nucleotides are used. Adenosine can be replaced by N^1^-methyladenosine (m^1^A) or N^6^-methyladenosine (m^6^A), cytidine by 5-methylcytidine (m5C) and uridine by 5-methyluridine (m5U), 2-thiouridine (s2U), 5-methoxyuridine (5moU), pseudouridine (ψ) or N1-methylpseudouridine (m1ψ). As an additional benefit, m5C and ψ also increase translation efficiency. As mRNA gets recognized by its high uridine content, reducing uridine-rich regions through codon optimization is an additional tool to lower the immunogenicity of mRNA also in the absence of further base modifications [15,17,36].

The article "Designing biomaterials for the delivery of RNA therapeutics to stimulate bone healing" was published in 2021. Journal: Mater Today Bio.

Although chemical modifications and alterations of the different mRNA elements can improve translation efficiency and RNA stability to yield expression over several day [38,39], the biological half-life of mRNA is short compared to the process of bone healing, which takes weeks rather than days [40].To overcome this shortcoming, bone-substituting biomaterials can be used to yield a sustained delivery of RNA nanocomplexes. Thus, these biomaterials can be used as an additional tool to i) protect RNA from degradation, ii) act as a reservoir for sustained delivery of RNA nanocomplexes [38], and iii) prevent leakage of RNA nanocomplexes to ectopic sides, thereby providing better spatial control over the delivery.

In contrast to strategies for RNA complexation and delivery, research on the incorporation of delivery-competent mRNA into biomaterials is still in its infancy. Therefore, this review will provide a comprehensive overview of the use of biomaterials as a delivery platform for RNA nanocomplexes within the overall context of bone regeneration. By reviewing current approaches toward ​the fabrication of RNA-delivering biomaterials for bone regeneration, we will specifically focus on:

• strategies for loading RNA nanocomplexes into biomaterial carriers;
• degradation of biomaterial carriers designed for RNA delivery;
• spatiotemporal control of biomaterial-based RNA delivery.

The timely orchestration of biochemical signals is crucial for successful tissue regeneration [41]. Therefore, we aim to correlate the design of RNA-delivering biomaterials to the various stages of bone healing. Moreover, we will also discuss the clinical handling of these biomaterials. Overall, by highlighting the various challenges associated with RNA delivery from multiple angles, we aim to create a holistic view to guide biomaterial design for RNA nanocomplex delivery.

The article "Designing biomaterials for the delivery of RNA therapeutics to stimulate bone healing" was published in 2021. Journal: Mater Today Bio.

## 2 Biology of bone healing

Bone defects can result from, for example, trauma, aging, degenerative bone diseases or tumor resection. In embryonic bone development, there are two distinct ossification pathways, which are intramembranous and endochondral ossification. During intramembranous ossification, mesenchymal stem cells directly differentiate into bone-forming cells, whereas endochondral ossification involves the formation of a cartilaginous intermediate (callus) which is mineralized in subsequent stages of ossification [42,43]. For this review, we will focus on endochondral ossification, as most bone defects heal via this pathway [40]. In the following section, we will provide a brief overview of this process and focus on relevant signaling molecules as possible targets for RNA therapeutics.

Bone healing involves several stages (Fig. 2). The initial phase of bone healing involves the formation of a hematoma and subsequent initiation of an inflammatory response [44]. Mesenchymal stem cells (MSCs) and chondrocytes are recruited to the tissue damage, the latter secreting collagen and other matrix proteins which form a soft callus [42,45]. This cartilaginous structure stabilizes the fracture and serves as a template for new bone formation [46]. Concurrently, primary new blood vessels form to secure blood supply to the new-forming tissue [1,45]. A dense fibrous tissue is formed within the soft callus and chondrocytes become hypertrophic while MSCs differentiate into osteoblasts [43,45]. Mineralization of the fibrous tissue results in calcified cartilage (hard callus) [1,43]. Finally, the bony callus undergoes remodeling. Osteoclasts resorb the mineralized cartilage, while osteoblasts deposit mature lamellar bone [42,44]. The primary vasculature regresses and is replaced by mature blood vessels [1]. During this phase of bone remodeling, the processes of matrix degradation and bone formation, which rely on osteoclasts and osteoblast, respectively, need to be finely balanced [42,44]. Although the initial stages of bone healing take about 1–2 months in humans, full remodeling of regenerated bone may take several years depending on biomechanical conditions [1].

**Fig. 2:** **Stages of bone healing and involved signaling molecules.** Stages of bone healing and main cell types involved are depicted in the top row. The expression of signaling molecules is shown in continuous lines for the different stages of bone healing. Dashed lines represent time spans where expression profiles vary between the various studies. The time scale of regeneration is based on bone healing in rodents. Abbreviations: IL, interleukin; TNF-α, tumor necrosis factor alpha; PDGFs: platelet-derived growth factors; TGF-β, transforming growth factor beta; BMP, bone morphogenetic protein; Wnt, proteins involved in Wnt signaling; VEGF, vascular endothelial growth factor; Ang, angiopoietin; MMP, matrix metalloproteinase; Dkk3, Dickkopf-related protein 3. Data based on [1,40,45,77,123,129,130].

The article "Designing biomaterials for the delivery of RNA therapeutics to stimulate bone healing" was published in 2021. Journal: Mater Today Bio.

### 2.1 Signaling molecules orchestrating bone healing

#### 2.1.1 mRNA targets

mRNA encoding osteogenic proteins has the potential to directly promote cell differentiation, matrix deposition, and vascularization. The most commonly studied osteogenic proteins for delivery in proteinaceous form belong to the family of BMPs, which are capable of inducing bone formation (especially BMP-2, BMP-6, BMP-7, and BMP-9) [47,48]. Notably, approaches aimed at facilitating the delivery of osteogenic mRNA from biomaterials as an alternative to biomaterial-based growth factor delivery have also mainly focused on BMP-2 (Table 2), although other factors involved in bone regeneration (see Fig. 2) might also act as potential mRNA target. So far, biomaterial-based delivery of mRNA coding for BMP-2 has been tested using fibrin [9,49], collagen [[50], [51], [52], [53]], and calcium phosphate [49] carriers. However, these biomaterial carriers were not specifically designed for this purpose and do not offer strong control over spatiotemporal delivery characteristics.

**Table 2:** Overview of studies on biomaterial-based RNA delivery.

Biomaterial	RNA	Complexation agent	Complex size (nm)	Complex charge (mV)	Loading mechanism	Release 24 ​h (%)^a^	Release 72 ​h (%)^a^	Release 7 d (%)^a^	Release 14 d (%)^a^	Release 21 d (%)^a^	Transfection efficacy	Ref
**Biomaterial-based mRNA delivery**												
Biphasic calcium phosphate granules	FITC-hBMP2-cmRNA	Lipoplexes (DreamFect Gold)	–	–	Diffusion	42	62	92	–	–	MetLuc mRNA expression: 10× increase (24–120 ​h)	[49]
Fibrin gel	FITC-hBMP2-cmRNA	Lipoplexes (DreamFect Gold)	–	–	Incorporation	20	34	43	–	–	MetLuc mRNA expression: 10× increase (24–120 ​h)	
Alginate hydrogel	Cy3-hGLuc-mRNA	Lipoplexes (GenaxxoFect)	–	–	Incorporation	28	52	66	72	79	N/A	[97]
Chitosan hydrogel	Cy3-hGLuc-mRNA	Lipoplexes (GenaxxoFect)	–	–	Incorporation	15	28	32	36	42	N/A	
Alginate-Chitosan hydrogel	Cy3-hGLuc-mRNA	Lipoplexes (GenaxxoFect)	–	–	Incorporation	29	50	59	62	69	Luminescence: 15,000× higher (24 ​h), 4× higher (7 d)	
**Biomaterial-based siRNA delivery**												
Methacrylated glycol chitosan hydrogel	siNoggin	Sterosome	155	33	Incorporation	5	14	31	58	–	Noggin expression: 40% decrease (3 d), 45% decrease (7 d)	[104]
Chitosan sponge	siCkip-1 or siCkip-1 ​+ ​siFlt-1	Lipofectamine	80	–	Diffusion	–	5	12	44	70	Cy5-siCkip-1: 95% positive cells, FAM-siFlt-1: 90% positive cells (24 ​h)	[93]
Polydopamine-coated PLGA film	siGFP	Lipidoids	60	–	Covalent	–	–	–	–	<5	GFP expression: 70% decrease (48 ​h)	[111]
Mono(2-acryloyloxyethyl) succinate–modified DEX hydrogel	siGFP (thiolated)	None	–	–	Covalent	30	52	76	82	–	No transfection	[116]
Mono(2-acryloyloxyethyl) succinate–modified DEX hydrogel	siGFP (methacrylated)	None	–	–	Covalent	45	60	78	92	–	GFP expression: 40% decrease (24 ​h), 50% decrease (48 ​h), 30% decrease (7 d)	
Double cross-linked PEG hydrogel (15 w/v%)	siGFP	PEI (no UV)	–	–	Incorporation	–	7	25	40	54	N/A	[99]
		PEI (with UV)	–	–	Incorporation	–	10	56	82	90	N/A	
Double cross-linked PEG hydrogel (22.5 w/v%)	siGFP	PEI (no UV)	–	–	Incorporation	–	1	3	8	18	GFP expression: releasant D2: 80% decrease, D6: 30% decrease, D14: 10% decrease (24 ​h culture)	
		PEI (with UV)	–	–	Incorporation	–	10	30	48	60	GFP expression: releasant D2: 90% decrease, D6: 50% decrease, D14: 25% decrease (24 ​h culture)	
Mono(2-acryloyloxyethyl) succinate–modified DEX hydrogel	siGFP	Branched PEI	–	–	Incorporation	–	8	10	20	48	N/A	[105]
Gelatin-PEG gel cross-linked with oPNMA anhydrin	siLuc	Low MW branched PEI	200	30	Diffusion	–	41	63	78	94	Luciferase expression: 20% decrease (72 ​h)	[95]
		Tyrosine-modified PEI	330	17	Diffusion	–	31	31	31	31	Luciferase expression: 20% decrease (72 ​h)	
		Lipopolyplexes	165	−3	Diffusion	–	16	41	56	75	Luciferase expression: 20% decrease (72 ​h)	
Gelatin-PEG gel cross-linked with oPDNMA anhydrin	siLuc	Low MW branched PEI	200	30	Diffusion	–	78	94	94	94	Luciferase expression: 15% decrease (72 ​h)	
		Tyrosine-modified PEI	330	17	Diffusion	–	31	31	31	31	Luciferase expression: 35% decrease (72 ​h)	
		Lipopolyplexes	165	−3	Diffusion	–	69	81	81	81	Luciferase expression: 5% decrease (72 ​h)	
PNIPAM-PEG-PNIPAM hydrogel	Fluc-siRNA	PNIPAM-PEG-PDMAEMA polyplexes	120–160 (at 37°C)	7 (at 37°C)	Incorporation	19	80	–	–	–	Luciferase expression: ∼25% decrease (24 ​h) with releasants of different time points	[101]
Methacrylated PEG with PEG-SH	FITC-cyclophilin B siRNA	PEI	–	–	Incorporation	10	20	28	58	–	GFP expression: 15% decrease (24 ​h)	[64]
Acrylated PEG with PEG-SH	FITC-cyclophilin B siRNA	PEI	–	–	Incorporation	8	13	19	30	41	GFP expression: 90% decrease (24 ​h); Noggin expression: 25% decrease (7 d), 65% decrease (14 d), 30% decrease (28 d)	
Dextran-HEMA hydrogel (8 w/w%)	FITC-cyclophilin B siRNA	Linear PEI (5 v/v% to gel)	–	–	Covalent	38	52	74	–	–	N/A	[110]
		Linear PEI (10 v/v% to gel)	–	–	Covalent	20	30	58	–	–	N/A	
Dextran-HEMA hydrogel (12 w/w%)	FITC-cyclophilin B siRNA	Linear PEI (5 v/v% to gel)	–	–	Covalent	32	43	54	80	–	siGFP: 90% decrease (3 d), 60% decrease (7 d)	
		Linear PEI (10 v/v% to gel)	–	–	Covalent	18	30	44	72	–	siGFP: 30% decrease (3 d), 25% decrease (7 d)	
Fibrin hydrogel	Alexa488-siRNA	Lipofectamine	120–160	Positive	Diffusion	70	80	–	–	–	Alexa488-siRNA: 98% positive cells (48 ​h)	[65]
PEG-b-poly(lactide)-*b*-dimethacrylate hydrogel	FAM-labeled NC-siRNA	DMAEMA-PAA-BMA polyplexes	30	14 (without siRNA)	Incorporation	23	47	60	70	75	Wwp1 expression: 80% decrease (3 d), 70% decrease (10 d), 50% decrease (12 d)	[128]
Alkali-treated titanium scaffold	Cy3-cmsiMIR31HG	Chitosan (no particles)	–	–	Diffusion	78	88	96	–	–	MIR31HG expression: 60% decrease (24 ​h), 40% decrease (7 d)	[92]
**Biomaterial-based miRNA delivery**												
PLLA scaffold and PLGA (64 ​kDa) microspheres	miR-26a	Hyperbranched polyester with PEI and PEG	120	13	Diffusion	30	34	38	52	56	N/A	[94]
		Linear polyester with PEI and PEG	160	7	Diffusion	30	34	44	53	61	N/A	
PLLA scaffold and PLGA (6.5 ​kDa) microspheres	miR-26a	Hyperbranched polyester with PEI and PEG	120	13	Diffusion	55	62	67	75	79	Cy3-miR-26a 40% positive cells (48 ​h)	
		Linear polyester with PEI and PEG	160	7	Diffusion	57	68	74	81	83	Cy3-miR-26a 20% positive cells (48 ​h)	
Chitosan/beta-glycerol-phosphate hydrogel	AntimiR-138	Chitosan	150	20	Incorporation	18	32	38	43	45	N/A	[98]
O-carboxymethyl chitosan matrix	FAM-labeled miR-21	APM polymeric nanocapsules	25	15	Incorporation	52	62	–	–	–	60% transfected cells (48 ​h)	[103]
		Lipofectamine	40	54	Incorporation	58	68	–	–	–	17% transfected cells (48 ​h)	
Poly(citrate-siloxane) - poly(ε-caprolactone)	miR-5106	PCEE	–	–	Incorporation	36	–	–	–	–	miR-5106 expression: 4.5-fold higher (7 d) and 7-fold higher (14 d) compared to PCL scaffold	[102]
PEG–PLGA–PNIPAM colloidal gel	miR-222	MSNs	200	3	Incorporation	–	20	42	60	71	N/A	[100]
PEG-gelatin-norborene hydrogel (10 w/v%)	Block-iT oligonucleotide	Lipofectamine	460	−14	Incorporation	1	23	70	–	–	97% positive cells (24 ​h)	[106]
		PEI 40 ​kDa	340	−7	Incorporation	9	41	76	–	–	77% positive cells (24 ​h)	
		PEI 4 ​kDa	220	−1	Incorporation	15	32	77	–	–	79% positive cells (24 ​h)	

Abbreviations: oPNMA, maleic anhydride–containing oligomeric cross-linker; oPDNMA, acrylamide anhydride–containing oligomeric cross-linker; PLLA, poly-l-lactic acid; PLGA, poly(lactic-co-glycolic acid); DEX, dextran; HEMA, hydroxyl ethyl methacrylate; PEG, polyethyleneglycol; PNIPAM, b-poly(N-isopropylacrylamide); PDMAEMA, poly(2–26 dimethylaminoethyl methacrylate); PEI, polyethyleneimine; DMAEMA, dimethylaminoethyl methacrylate; PAA, propylacrylic acid; BMA, butyl methacrylate; APM, N-(3-Aminopropyl)methacrylamide; PCEE, polycitrate-polyethyleneglycol-polyethyleneimine; MSNs, mesoporous silica nanoparticles; MW, molecular weight; Diffusion, diffusional post-loading; Covalent, covalent bonding.

a Only studies investigating release rates of RNA complexes from biomaterials were included. When values were not reported in the text, presented numbers were derived from graphs.

The article "Designing biomaterials for the delivery of RNA therapeutics to stimulate bone healing" was published in 2021. Journal: Mater Today Bio.

Besides direct stimulation of bone healing via growth factors, immunomodulation has recently emerged as an alternative approach to promote bone healing. M1 polarized macrophages are pro-inflammatory, whereas polarization toward ​the M2 phenotype is considered anti-inflammatory and tissue-regenerative [54]. Indeed, *in vitro* studies have shown that transition from pro-inflammatory M1 macrophages to regenerative M2 macrophages enhances the osteogenic potential of pre-osteoblasts [55,56]. However, it should be realized that transient pro-inflammatory signaling is necessary to achieve bone regeneration [55] and to potentiate the osteogenic effect of BMP-2 [57]. Biomaterial-based immunomodulation strategies to stimulate bone healing published so far include the use of NEMO-binding domain peptide to block B cell activation [58], biomimetic anti-inflammatory nanocapsules capturing pro-inflammatory cytokines [59], and gene delivery of interleukin 1 receptor antagonist [60].

#### 2.1.2 siRNA targets

In addition to mRNA-dependent expression of growth factors, it is also possible to induce therapeutic effects by downregulation of inhibitory protein expression using siRNAs [15]. Hereafter, we shortly highlight the most prominent inhibitors, focusing on well-researched molecules acting as BMP antagonists.

Chordin, Noggin and Gremlin are well-known antagonists of BMPs such as BMP-2 and BMP-7 ​and are therefore interesting targets to enhance bone regeneration [47]. Downregulating the expression of Chordin with siRNA was shown to increase osteogenic differentiation and bone regeneration *in vitro* and *in vivo* [[61], [62], [63]]. Similarly, silencing of Noggin using siRNA did promote osteogenic differentiation *in vitro* and *in vivo* [[64], [65], [66]]. However, simultaneous supplementation with proteinaceous BMP-2 is needed since only silencing Noggin showed no effect on osteogenic differentiation *in vitro* [61]. Similarly, downregulation of Gremlin was found to improve osteogenic differentiation. Yet, for Gremlin the experiments were only conducted in the presence of BMP-2, so it is not clear to which extent downregulation alone would also exert an effect [63].

As mentioned previously, bone regeneration can also be triggered by immunomodulation. A pro-inflammatory environment inhibits osteogenic differentiation and promotes MSC apoptosis [67,68], and neutralization of pro-inflammatory cytokines has been shown to promote bone regeneration *in vivo* [59,68]. Similarly, downregulation of these cytokines using siRNA may be beneficial for bone healing.

The article "Designing biomaterials for the delivery of RNA therapeutics to stimulate bone healing" was published in 2021. Journal: Mater Today Bio.

#### 2.1.3 miRNA targets

Although research on biomaterial-based RNA delivery has mainly focused on mRNA and siRNA, several studies have demonstrated promising *in vitro* and *in vivo* results for the application of miRNAs to stimulate bone healing [69]. A plethora of miRNAs are involved in bone formation and homeostasis by targeting negative regulators of osteogenesis or positive regulators of osteoclastogenesis [25,70]. Moreover, differentially expressed miRNAs have been identified for several skeletal diseases, such as osteoporosis, osteoarthritis and bone non-union [71,72]. The majority of these miRNAs were found to be overexpressed under diseased conditions, thereby affecting osteoblast or osteoclast activity. Interestingly, miRNAs related to bone formation were mostly targeting the expression of transcription factor RUNX-2 or SP7 (also known as osterix) [71,73] and may serve as targets to promote bone regeneration. Both transcription factors are important for the differentiation of bone marrow stromal cells to pre-osteoblasts, ​and pre-osteoblasts to mature osteoblasts, respectively ​[74]. In addition, BMP-2 expression and its respective receptor BMPR-2 were identified as other common targets of differentially expressed miRNAs [71]. A comprehensive overview of miRNAs involved in bone homeostasis and disease can be found elsewhere [25,71,72,75,76].

## 3 Spatiotemporal control over RNA delivery

Research on biomaterial-based RNA delivery is still in its infancy and only few published results are available (Table 2). Nevertheless, we argue that early identification of the main hurdles toward ​translation of RNA-containing biomaterials into the clinic will prevent loss of time and expenses on the development of strategies that will not be translatable. Therefore, an overview of design criteria is provided in Fig. 3. Currently, research on RNA delivery mainly focuses on the design of complexation agents to protect the RNA and facilitate cellular internalization. In contrast, biomaterial carriers are not yet specifically designed to achieve spatial and temporal control over the delivery of RNA formulations. In the following section, we will discuss these two key aspects of RNA delivery in more detail.

**Fig. 3:** Design criteria for RNA-delivering biomaterials.

### 3.1 Temporal control

As illustrated in Fig. 2, many signaling molecules are only present at a distinct phase during bone healing. BMP-2, for example, shows a biphasic expression pattern with a first peak around Day 3 and a second one between Days 14 and 21 [77]. However, studies testing biomaterial-based delivery of BMP-2-encoding mRNA show mRNA release as of Day 1 [9,49]. So far, it is not known whether the timing or duration of BMP-2 mRNA delivery has an impact on bone healing. In contrast, temporal control is clearly of importance in dual delivery systems of proteinaceous growth factors. Several growth factors, including TGF-β1 and PDGF, have been found to inhibit BMP-2-induced osteogenic differentiation when delivered at the wrong time point (reviewed in Refs. [78,79]). However, such temporal control is currently not taken into account for the design of current biomaterials for RNA delivery.

The article "Designing biomaterials for the delivery of RNA therapeutics to stimulate bone healing" was published in 2021. Journal: Mater Today Bio.

For biomaterial-based delivery platforms, the rate and type of degradation is key to regulating the release kinetics of embedded bioactive molecules. However, such delivery platforms face a twofold challenge. On the one hand, the delivery kinetics should match the biological temporal sequence of growth factor orchestration [80]. On the other hand, the rate of biomaterial degradation should correspond with the rate of ingrowing tissue ​while still providing enough mechanical support [10,81]. Particular challenges arise when the desired kinetics of biomolecule delivery and biomaterial degradation are out-of-phase, for example, when biomolecule release should proceed faster than biomaterial carrier degradation. Numerous factors influence the mechanical properties and degradation characteristics of biomaterials, and the interested reader is referred to other reviews discussing this topic [80,82].

### 3.2 Spatial control

The serious clinical side effects observed for BMP-2 delivery from biomaterials [[83], [84], [85]] showcase the importance of spatial control over the delivery of bioactive compounds. Here, lack of spatial control (leakage) and rapid degradation of BMP-2 were compensated for by loading excessive amounts of this therapeutic protein, locally leading to about one million times higher protein concentrations than physiological conditions [13]. The combination of these supraphysiological amounts and off-target effects due to leakage caused life-threatening side effects, including osteolysis, dysphagia, inflammation of the nerve root and associated neurological deficits [[11], [12], [13]].

Biomaterials can act as a storage for biomolecules, thereby retaining the bioactive compound at the application site and limiting leakage to ectopic sites. Spatial control over the delivery of bioactive compounds also allows to lower the amount of loaded cargo, which further reduces the risk of adverse events [24,80].

The article "Designing biomaterials for the delivery of RNA therapeutics to stimulate bone healing" was published in 2021. Journal: Mater Today Bio.

## 4 Modulating RNA delivery from biomaterials

Successful delivery of RNA requires three key aspects:

1) **RNA protection**: RNA needs to be protected from premature degradation and maintain its bioactivity upon delivery [18,37]. For his purpose, chemically modified RNAs (cmRNAs) and complexation agents have been developed, which have been extensively reviewed elsewhere [15,17,18,86]. However, biomaterials can also be exploited to protect encapsulated RNA from degradation by nucleases and prevent recognition by the immune system [87]. For this application, the biomaterial carrier must not disturb the interactions between RNA and the complexation agent, ​since this would lead to premature decomplexation (see Section 4.4 on RNA decomplexation).
2) **RNA dosing:** RNA dosing should be sufficiently low to minimize side effects ​but sufficiently high to elicit the desired therapeutic effect. However, studies on RNA dosing are still scarce. The cellular uptake of RNA relies on biochemical interactions of the RNA formulation with the cell membrane and subsequent endocytosis. Once internalized, the RNA needs to escape the endosome before it is degraded by the acidic environment and hydrolases. Subsequently, RNA complexes should be unpacked to facilitate access of the RNA to the relevant enzyme complexes (i.e., ribosomes in the case of mRNA and RISC complex in the case of siRNA and miRNA) [15] ​[[88], [89], [90]].
3) **RNA delivery kinetics:** Similarly to growth factors, RNA should be delivered in a biologically meaningful time frame, that is, the duration of release and amount of delivered RNA should match the bone healing process as closely as possible to attain optimal therapeutic efficacy [41]. The required release duration depends on the targeted biomolecule (see Fig. 2). In this context, biomaterials can act as a reservoir to achieve temporal control over the delivery [91]. Delivery kinetics are mainly determined by i) the loading mechanism of RNA complexes to a biomaterial, ii) the degradation of the biomaterial matrix and iii) the interactions between RNA complexes and the biomaterial.

### 4.1 RNA loading strategies

Based on the current literature on biomaterial-based RNA delivery (Table 2), three main strategies for loading complexed RNA (in)to biomaterials can be discerned, namely i) diffusional post-loading after material fabrication, ii) incorporation into the material and iii) covalent binding after fabrication (Fig. 4).

**Fig. 4:** **Loading of RNA into biomaterial carriers.** Schematic illustration of loading strategies for RNA into biomaterials. Left: mRNA, miRNA or siRNA is complexed with a complexation agent before loading into the biomaterial. Right: Double-stranded siRNA is modified with linker molecules before covalent bonding to the biomaterial.

The article "Designing biomaterials for the delivery of RNA therapeutics to stimulate bone healing" was published in 2021. Journal: Mater Today Bio.

#### 4.1.1 Diffusional post-loading of RNA onto biomaterials

Diffusional post-loading is achieved by impregnating or soaking a pre-made biomaterial after fabrication with an RNA complex-containing solution. Depending on the nanoscale porosity of the biomaterial, the RNA complexes will either penetrate the biomaterial or adsorb onto its surface. This simple loading method has been used for a variety of biomaterials, including metals [92], polymeric scaffolds [65,[93], [94], [95]], and calcium phosphates [49].

For example, Huang et al. [92] soaked a titanium scaffold with a porous surface structure in a chitosan-siRNA solution followed by a washing and drying step. The authors showed siRNA loading efficacies of up to about 70% (after 8 ​h soaking) and a homogenous distribution of siRNA over the titanium surface. However, after 24 ​h, already 80% of siRNA was released. Despite this rapid release of siRNA, gene silencing was sustained for 7 days *in vitro*.

In contrast, a more prolonged release using diffusional post-loading was achieved by Balmayor et al., who adsorbed mRNA lipoplexes to porous biphasic calcium phosphate (BCP) granules followed by lyophilization. After 24 ​h, 42% of loaded mRNA was released from the BCP granules, and release was sustained for 7 days. The BCP granules contained 60% hydroxyapatite (HA), a material which has also been used for complexation of RNA [96]. This material selection might have contributed to the strong retention of mRNA observed in this study. The same study also showed that incorporation of the mRNA lipoplexes within a fibrin hydrogel resulted in slower release (20% released after 24 ​h) compared to diffusional post-loading on BCP granules, confirming that incorporation of mRNA slows down RNA delivery kinetics as compared to post-diffusional post-loading. Both systems showed successful transfection of cells using *Metridia* luciferase (MetLuc) mRNA over 5 days.

In general, it can be concluded that diffusional post-loading is the simplest loading strategy which enables efficient loading of mRNA onto biomaterials. However, release kinetics are difficult to control because the RNA complexes are associated with the biomaterial rather weakly by non-covalent interactions, resulting in burst-type release patterns and limited control over long-term delivery kinetics.

#### 4.1.2 Incorporation of RNA into biomaterials

Incorporation of RNA complexes into biomaterials can be achieved by adding RNA complexes to the biomaterial before the formation of the final biomaterial matrix. This approach is most often adopted for hydrogels, where the RNA complexes are mixed into the polymer solution before cross-linking the gel. So far, most studies investigated hydrogels made of natural [49,97,98] or synthetic [62,64,[99], [100], [101], [102]] polymers or a mixture thereof [[103], [104], [105], [106]], but RNA complexes have also been successfully mixed into inorganic HA cements [107]. Compared to diffusional post-loading, where the complexes are loosely associated with the material, this method usually leads to stronger retention of RNA complexes and thus to release kinetics that depend on degradation of the polymer matrix.

The article "Designing biomaterials for the delivery of RNA therapeutics to stimulate bone healing" was published in 2021. Journal: Mater Today Bio.

Steinle et al. [97] used hydrogels made of the natural polymers alginate or chitosan or a mixture thereof ​and incorporated RNA lipoplexes into the hydrogels. For all three types of gels, a sustained mRNA release of up to 21 days was accomplished. Alginate gels showed the fastest release kinetics with 79% of mRNA released after 21 days compared to 69% for alginate-chitosan gels and 42% for chitosan gels. The authors attributed these differences to the positive charge of chitosan and negative charge of alginate, thereby favoring repulsion or attraction of the mRNA lipoplexes, respectively. Indeed, interactions between biomaterial and RNA complexes are a key factor for modulating release rates, as we will discuss in Section 4.3.

Synthetic polymers offer the specific opportunity to tune release rates by modifying polyplex behavior or network formation characteristics of the hydrogel matrix. Fliervoet et al. [101] used triblock polymers of b-poly(N-isopropylacrylamide) (PNIPAM), polyethyleneglycol (PEG) and poly(2-26 dimethylaminoethyl methacrylate) (PDMAEMA) to produce thermosensitive siRNA polyplexes (PNIPAM-PEG-PDMAEMA) and a thermosensitive hydrogel (PNIPAM-PEG-PNIPAM). Although they successfully demonstrated thermosensitive behavior of both the polyplexes upon heating from 10°C to 37°C, the benefit of such a system may be questionable in view of the constant body temperature. The thermosensitive hydrogels allowed for *in situ* gelation, and the authors demonstrated injectability of the gel through a 23G needle (inner diameter ca. 0.4 ​mm), albeit without specification of the temperature. Their system showed a relatively fast delivery under physiological conditions (37°C) since 80% of siRNA complexes were released after 3 days. Considering the relatively constant release between the various time points, the authors suggested that the release was governed by hydrogel degradation rather than by diffusion of siRNA complexes.

Summarizing, incorporation of RNA within a biomaterial matrix can improve control over RNA delivery kinetics. Sustained delivery of RNA has been shown for up to 21 days. Depending on the hydrogel mesh and size of the RNA complex, the release of incorporated RNA complexes is governed by diffusion, hydrogel swelling and/or network degradation. Polymer concentration, molecular weight (MW), cross-linking density, and resultant mesh size are the main factors influencing the release kinetics [47,108]. If the hydrogel possesses a mesh size bigger than the incorporated complexes, the release is governed by diffusion which can be modulated by network–complex interactions. In this case, the system will display release characteristics similar to diffusional postloading. If the mesh size is comparable to the size of the complexes, diffusion is sterically hindered, which significantly slows down complex diffusion. However, diffusivity of RNA complexes can be increased again upon swelling of the network due to the enlargement of the mesh size. Moreover, mechanical deformation can also increase the number of released complexes by increasing convective flow and 'squeezing' the cargo out of the hydrogel. In hydrogels with very small mesh size, the RNA complexes are entrapped and can only be released upon network degradation [91,108,109]. Finally, it should be stressed that the mesh size of a degrading hydrogel is time-dependent for polymer meshes degrading via bulk erosion (see below). In those cases, the mesh size will increase with advanced degradation [109].

The article "Designing biomaterials for the delivery of RNA therapeutics to stimulate bone healing" was published in 2021. Journal: Mater Today Bio.

#### 4.1.3 RNA loading by covalent attachment

The third main loading strategy involves covalent attachment of RNA complexes to biomaterials after their fabrication using linker molecules. Although this approach theoretically allows for improved control over RNA release kinetics compared to diffusional postloading or incorporation, this loading method requires additional modification steps, such as the synthesis of suitable linker molecules. So far, only two groups have investigated covalent binding for biomaterial-based RNA delivery.

Nguyen et al. [110] used a dextran-methacrylate hydrogel and methacrylate-containing polyethyleneimine (PEI) to form covalent ester cross-links between siRNA-PEI complexes and the hydrogel. Slower release was observed at higher contents of the complexation agent and higher polymer content in the gel. For the gel with low polymer content, all siRNA was released after 9 days irrespective of the content of complexation agent since the gel was then completely degraded. At higher polymer contents, the biomaterial carrier degraded at a slower rate which resulted in more sustained siRNA delivery (complete release after 17 days). The authors concluded that siRNA was released from the gels by a combination of diffusion (initial burst) and hydrogel degradation (at later time points).

The article "Designing biomaterials for the delivery of RNA therapeutics to stimulate bone healing" was published in 2021. Journal: Mater Today Bio.

Shin et al. [111] aimed at higher transfection efficiency of attached cells by localizing RNA complexes to the material surface. For this purpose, a very stable immobilization of siRNA was achieved by using polydopamine-coated poly(lactic-*co*-glycolic acid) (PLGA) films and siRNA complexed with lipidoids. Less than 5% of siRNA was released from the PLGA films after 21 days, illustrating the strong retention capacity enabled by covalent catechol-amine interactions between catechol groups of polydopamine and amines of the siRNA-lipidoids. Interestingly, successful cellular transfection was already observed after 2 days of culture. Moreover, transfection efficacy of substrate-bound siRNA-lipidoids was higher compared to suspended siRNA-lipidoids (68.9 ​± ​3.7% vs. 48.8 ​± ​6.3% for siGFP, ​and 26.8 ​± ​3.5% vs. 38.3 ​± ​5.5% for siGAPDH), which was attributed to increased cell-siRNA contact. These results also demonstrate that very high effective siRNA concentrations can be achieved through local immobilization.

Generally, for covalently linked systems, the RNA release rate is defined by the cleavage rate of the linkage [109]. Surprisingly, release rates of RNA complexes were not substantially lower upon covalent linkage compared to incorporation, except when catechol-amine bonds were formed. This linking method also successfully prevented the initial burst release [111]. Ester bond cleavage occurs by spontaneous hydrolysis or through enzymatic cleavage by the ubiquitously present esterases in the cell [112]. Disulfide bond reduction uses the glutathione cycle and associated enzymes [113,114]. Catechol-amine bonds are formed between primary amines and catechol groups. Those very strong C-N bonds are harnessed for the development of medical adhesives. Bond formation is promoted by a low pKa value of the primary amine and a neutral or mildly acidic pH [115]. Thus, bond cleavage is likely to occur under alkaline conditions, similar to ester bonds. Importantly, chemical modification of RNA for covalent bonding may impede cell internalization as observed by Nguyen et al. [116] (see Section 4.3). Therefore, cleavage of covalently linked RNA should ideally release the RNA in unmodified form.

### 4.2 Biomaterial matrix degradation

Biomaterial matrix degradation is an established tool to modulate release kinetics for any sort of cargo. Consequently, biomaterial degradation mechanisms have been extensively studied and excellent reviews on this topic are available elsewhere [80,108,117]. Matrix degradation is particularly crucial for kinetics of RNA delivery when RNA complexes are either incorporated into the biomaterial or tightly linked to the biomaterial, ​either by non-cleavable covalent bonds or by strong electrostatic interactions upon diffusional post-loading (see also Section 4.3).

The article "Designing biomaterials for the delivery of RNA therapeutics to stimulate bone healing" was published in 2021. Journal: Mater Today Bio.

Generally, degradation of biomaterials can either proceed heterogeneously from outside to inside ​or homogeneously throughout the entire bulk material. The biomaterial permeability for the degrading agent (e.g., enzymes or solvent) is strongly determining the nature of the degradation mechanism. If this permeability is limited, biomaterials will degrade mainly at the edges, resulting in surface erosion [80,108]. During this process, biomaterial fragments or monomers can be detached from the bulk material [118,119]. On the other hand, highly permeable materials show bulk degradation. This uniform degradation increases the porosity of the biomaterial, which leads to biomaterial instability and allows more rapid diffusion of the cargo as shown by the mathematic model of Chen et al. [118].

#### 4.2.1 Degradation of hydrogel matrices

RNA delivery from hydrogels is often enabled by incorporation of the RNA complexes into the biomaterial (see Section 4.1.2), which offers the possibility to tune the release kinetics of RNA complexes by modifying the degradation behavior of the hydrogel. Natural polymers such as collagen, gelatin or hyaluronan degrade by enzymatic cleavage of the polymer chains, whereas most synthetic polymers such as polyesters undergo spontaneous hydrolysis of intra- or inter-molecular bonds [108]. The most important parameters influencing the degradation rate of hydrogels are the MW of the polymer, polymer composition and cross-linking density of the hydrogel, surface/volume ratio, porosity of the hydrogel and diffusivity of solvents and solutes [47,108].

Hydrogel degradation can also be induced using external triggers, such as light, temperature or pH changes. For example, Huynh et al. fabricated a dual cross-linked PEG hydrogel with and without ultraviolet (UV)-degradable cross-linkers for on-demand RNA delivery [99]. The release of siRNA-PEI complexes was about twice as fast upon daily UV light exposure for 10 ​min compared to non-exposed gels (82% vs. 40% release after 14 days). The faster RNA release correlated well with the twofold faster degradation as observed for the UV-degradable hydrogels compared to the gels without UV-degradable cross-links. Although the UV light–triggered release may not be the most feasible option in terms of clinical handling due to limitations related to penetration depth and potential cross-linking of nucleobases, such on-demand delivery could offer the possibility for increasing the release at specific time points to match, for example, the biphasic expression pattern of BMP-2 (Fig. 2). On-demand drug delivery is heavily researched and reviewed elsewhere [[120], [121], [122]]. Although pH-responsive systems have not yet been used extensively to stimulate bone healing, such pH-responsive systems might offer specific advantages to support early stages of bone healing when hypoxic conditions during initial inflammation and early callus formation lead to locally reduced pH values in healing bone [42,123].

The article "Designing biomaterials for the delivery of RNA therapeutics to stimulate bone healing" was published in 2021. Journal: Mater Today Bio.

#### 4.2.2 Degradation of calcium phosphate–based materials

The degradation of calcium phosphates occurs via either passive chemical dissolution and/or active cell–mediated resorption [117]. Intrinsic factors determining the degradation kinetics of calcium phosphates include porosity, pore size, shape, surface-to-volume ratio, phase composition, crystallinity and inclusion of additional ions (doped calcium phosphates). Extrinsic factors influencing the degradation rate are pH, temperature, oxidative environment and enzymes [80,82,124].

Although calcium phosphate–based materials are widely used in clinical practice, only two studies have tested RNA delivery from these materials so far [49,107]. Utzinger et al. [107] incorporated PLGA microspheres containing cmRNA ​lipoplexes into a commercially available HA ​cement. HA cements are known to degrade relatively slowly (in the range of months to years) [125]. The PLGA microspheres not only served as a vehicle to deliver the cmRNA lipoplexes ​but also increased the porosity of the cement upon their hydrolytic degradation, which accelerated the degradation rate of cements [117,124]. Unfortunately, cmRNA release from PLGA microspheres and HA cement with microspheres was not directly assessed in this study. Nevertheless, comparable levels of protein expression were found for cells cultured on the microspheres-containing cement or with free microspheres after 48 ​h. Thereafter, a fast decrease in expression was observed for the cement compared to the microspheres only. The authors attribute this drop in protein expression to the slow erosion rate of HA cements and argued that transfection occurred mainly from surface-associated cmRNA lipoplexes.

### 4.3 Interactions between RNA complexes and biomaterials

#### 4.3.1 Biomaterial–RNA–complex interactions upon diffusional post-loading of RNA onto biomaterials

RNA complexes differ in size, surface charge and functional groups depending on the complexation agent used and the ratio between RNA and complexation agent (N/P ratio). The surface charge of RNA complexes and resulting electrostatic interactions with the biomaterial are particularly important in case of diffusional post-loading which depends on electrostatic interactions between RNA complexes and the biomaterial. In case of large RNA complexes or dense biomaterials, the complexes can only be retained at the biomaterial surface [4,126]. Usually, this scenario results in an initial burst phase due to relatively weak biomaterial–complex interactions with limited subsequent release. The charge of RNA complexes and biomaterials can also affect the distribution of RNA complexes throughout the biomaterial, as shown by Schwabe et al. [95] for negatively charged gelatin hydrogels and three different types of complexation agents (DPPC lipopolyplexes, low MW PEI and tyrosine-modified branched PEI). After diffusional post-loading, the positively charged low MW PEI and tyrosine-modified PEI-RNA-complexes were predominantly found on the gel surface. However, tyrosine-modified PEI-RNA-complexes, bearing a slightly lower charge, penetrated into the gel. In contrast, the almost neutral DPPC lipopolyplexes showed a homogenous distribution within the gel. Important to note, the lipopolyplexes were smaller (165 ​nm) compared to low MW PEI (200 ​nm) and tyrosine-modified PEI (330 ​nm) RNA complexes.

The article "Designing biomaterials for the delivery of RNA therapeutics to stimulate bone healing" was published in 2021. Journal: Mater Today Bio.

#### 4.3.2 Biomaterial–RNA–complex interactions upon incorporation of RNA into biomaterials

Upon incorporation of RNA complexes into biomaterials, release kinetics are modulated by the size of RNA complexes relative to the porosity or mesh size of the biomaterial as well as electrostatic interactions. Carthew et al. [106] investigated the effect of RNA complex size on their release rate using a PEG-gelatin-norborene hydrogel and RNA complexation with lipopolyplexes or PEI of different MW. After 24 ​h, release rates seemed to be inversely correlated to RNA complex size, with small low MW PEI (220 ​nm) showing the fastest release (15%) and large lipoplexes (460 ​nm) the slowest release (1%). Yet, after 7 days, similar amounts of oligonucleotides (70%–77%) were released for all three complexation agents, which might be caused by hydrogel swelling resulting in enlarged mesh size and increased diffusivity (especially for larger nanoparticles). However, the authors suggested that the differences in release were not only caused by the size of RNA complexes (lipoplexes ​> ​high MW PEI ​> ​low MW PEI) ​but also by their different charges. The most negatively charged lipoplexes (−14 ​mV) showed the slowest release compared to low MW PEI (−1 ​mV) and high MW PEI (−7 ​mV) RNA complexes, most likely due to their electrostatic with oppositely charged cationic gelatin (type A) in the hydrogel.

As illustrated previously, size and surface charge both play an important role in modulating the release rate of RNA complexes. However, as both parameters usually vary for different complexation agents, the respective contribution of either one is hard to determine. Also, relevant information may be missing since studies on biomaterial-based RNA delivery often do not report RNA complex characteristics.

The article "Designing biomaterials for the delivery of RNA therapeutics to stimulate bone healing" was published in 2021. Journal: Mater Today Bio.

#### 4.3.3 Biomaterial–RNA–complex interactions upon RNA loading by covalent attachment

Covalent bonding of RNA to a biomaterial is a very strong—and often irreversible—RNA-biomaterial interaction. However, chemical modification of RNA may impede its cellular internalization, as illustrated by Nguyen et al. [116], who covalently bound thiol end-modified siRNA to a hydrogel of mono (2-acryloyloxyethyl) succinate–modified dextran using hydrolytically cleavable β-thioether ester linkages. They demonstrated that the delivery of covalently bound siRNA was significantly slower compared to unbound siRNA lacking this thiol modification (30% vs 68% release after 24 ​h for bound and unbound siRNA, respectively). A plateau at 85% release was observed for unbound siRNA after 3 days. For covalently bound siRNA, a similar degree of release was only reached after 14 days. The authors suggested that the relatively rapid release observed for bound siRNA after 24 ​h was due to unbound siRNA in the hydrogel, whereas the subsequent release resulted from covalently bound siRNA. However, the released siRNA was unable to transfect cells, which was attributed to the presence of carboxyl end groups on the released siRNA. Therefore, the authors used an alternative chemistry to bind siRNA-methacrylate to the hydrogel based on ester and disulfide bonds. Upon reduction of the disulfide bonds or hydrolysis of the ester bonds, the siRNA would be released in a thiol- or hydroxyl-terminated form. In this system, similar but slightly faster release was observed with 45% after 24 ​h and 85% at Day 12. Successful cellular transfection was demonstrated, as reflected by gene silencing levels of 20%–70% depending on the amount of loaded siRNA and fetal bovine serum content of the medium.

Although the delivery of covalently linked RNA is mostly governed by the cleavage rate of covalent bonds, the release rate may again also be influenced by complex charge and size through electrostatic interactions and/or hindered diffusion. Importantly, release control via covalent binding requires that biomaterial degradation proceeds slower than bonds are cleaved ​since release kinetics might otherwise become influenced by matrix degradation as well.

### 4.4 RNA decomplexation

A specific requirement for RNA loading through incorporation into biomaterials involves the chemical compatibility between RNA complexes and the biomaterial matrix (except for naked siRNA). RNA complexes are typically formed through charge-driven non-covalent interaction of a positively charged complexation agent with the negatively charged oligonucleotide [17]. Evidently, RNA complexes should not be dissociated upon contact with the surrounding biomaterial. As discussed in Section 4.3, electrostatic interactions also occur between RNA complexes and the biomaterial, which can be used to increase complex retention. However, excessively strong complex–biomaterial interactions can lead to RNA decomplexation. Negatively charged biomaterials may compete with RNA for the positively charged complexation agents, while positively charged biomaterials can displace the complexation agent and directly bind to the negatively charged RNA. Indeed, RNA decomplexation has been observed by Schwabe et al. [95]. Using fluorescent labels on RNA and the complexation agent (PEI), they showed that the negatively charged RNA and the positively charged PEI were partially separated by the negatively charged gelatin hydrogels. Furthermore, they confirmed these results by an RNA displacement assay, which revealed that about 20% of RNA was released from the gelatin in complexed state.

The article "Designing biomaterials for the delivery of RNA therapeutics to stimulate bone healing" was published in 2021. Journal: Mater Today Bio.

### 4.5 RNA delivery *in vivo*

Delivery of RNA *in vivo* is confronted with the general challenge that any RNA complexes released into the blood stream will, to a major extent, be sequestered by the reticuloendothelial systems and thus accumulate in the liver. The incorporation of RNA complexes into locally applied biomaterials therefore offers the advantage that also the delivery of RNA is local. Ideally, only so much RNA complexes are released at a given point in time as can be locally taken up from cells in the immediate environment so that systemic exposure to the mRNA complexes is minimal.

So far, studies on RNA delivery from biomaterials have mostly been conducted in acellular conditions, especially when investigating release kinetics. Moreover, these quantifications of release kinetics are usually performed in simple phosphate-buffered saline (PBS). Although such acellular experiments provide a first impression of release kinetics, possible interactions with serum proteins and the extracellular matrix cannot be assessed. Similarly, traditional 2D *in vitro* experiments do not reflect the complexity of the physiological tissue environment and do not account for the effects of mechanical loading, perfusion, tissue mobility, and the presence of different cell types.

Three-dimensional (3D) *in vitro* models can recreate the physiological cell microenvironment more closely to provide more relevant biological information on cell matrix and cell–cell interactions [127] ​and the delivery of RNA complexes. For instance, Nguyen et al. [64] used a 3D cell culture models to assess siRNA delivery. However, delivery was still assessed indirectly by measuring the expression of target genes. Generally, studies directly investigating RNA delivery and distribution in 3D models are still lacking. Microfluidic chips and bioreactors will allow to study RNA delivery in 3D and under dynamic conditions. Furthermore, the effects of mechanical loading should be studied in more complex *in vitro* models, especially for RNA delivery from flexible biomaterials such as hydrogels.

The article "Designing biomaterials for the delivery of RNA therapeutics to stimulate bone healing" was published in 2021. Journal: Mater Today Bio.

Several studies have investigated RNA delivery kinetics *in vivo*, but so far, only endpoint measurements (e.g., amount of bone growth) have been reported instead of longitudinal monitoring of the release and distribution of RNA within tissues [53,93,98,103,111]. For the reliable quantification of RNA delivery kinetics *in vivo*, a major challenge relates to the penetration depth of the modality used to detect the labeled nanocomplexes in deep tissue layers. Bioluminescence and radiolabeling are potential options, although the latter labeling modality might negatively affect the biological activity of RNA through base mutation. Alternatively, conventional fluorescent labels have been used successfully by Wang et al. [128] to investigate the release of siRNA polyplexes from PEG-based hydrogels *in vivo*.

In summary, RNA delivery from biomaterials has mostly been studies in models which, by far, do not represent the complexity of the native tissue. Aspects such as perfusion, movement, interactions with extracellular matrix and cell type diversity may have a significant impact on RNA delivery *in vivo* ​but are not accounted for in current *in vitro* settings. Moreover, current *in vivo* tests mainly focus on demonstrating therapeutic efficacy rather than unraveling underlying mechanisms of RNA release and biodistribution.

## 5 Conclusion and future perspective

Problems related to local delivery of osteogenic GFs (mainly BMP-2) and clinical translation of delivery of osteogenic genes have prompted researcher to explore the opportunity of RNA therapy (including miRNA, siRNA and mRNA) for stimulation of bone healing. RNA delivery offers the possibility to transiently express any protein (including intracellular and transmembrane proteins) without the need for genomic integration by using the endogenous protein machinery of the cell. By providing a brief overview of the various stages in bone healing (Section 2), potential therapeutic RNA targets were reviewed. The biggest challenge for RNA delivery is the poor stability and transfection efficiency of naked RNA. Therefore, protection of RNA by complexation is crucial. Biomaterials can offer an additional tool to protect RNA complexes and allow for local delivery into bone defects. The importance of spatiotemporal control over RNA delivery was explained in Section 3 in the context of the biology of bone healing, followed by a comprehensive overview of biomaterial design tools (Section 4) that can be used to modulate RNA release characteristics, including i) the RNA loading strategy, ii) biomaterial degradation rate, and iii) interactions between biomaterial carriers and RNA complexes.

The article "Designing biomaterials for the delivery of RNA therapeutics to stimulate bone healing" was published in 2021. Journal: Mater Today Bio.

Biomaterial-based RNA delivery to stimulate bone healing is still in its exploratory phase. So far, the importance of spatial and temporal control of RNA-based therapeutics from biomaterials is hardly studied. To enable for spatial control over RNA delivery, injectable and *in situ* hardening materials are the most promising biomaterial candidates. These biomaterials allow for minimally invasive application (i.e., injection), which may reduce tissue damage, risk of infection and ultimately help to minimize the health burden for the patient. In this respect, retention of injectable materials at the injection site is crucial. Therefore, future studies should investigate *in vivo* biomaterial integrity, both directly after injection as well as on the long term after days to weeks of *in situ* delivery to avoid premature leakage of RNA complexes. To this end, self-healing biomaterials offer the opportunity to maintain biomaterial integrity even after destructive shearing upon injection through narrow needles.

Regarding temporal control of RNA-delivering biomaterials, it should be stressed that the optimal kinetics and durations of both biomaterial degradation and drug delivery are not yet known; optimal RNA doses remain to be determined as well. Therefore, dose–response studies, as commonly performed in pharmaceutical research, are required to deepen our understanding of biomaterial-induced RNA delivery.

Current biomaterials for RNA delivery do by far not reflect the complexity of the bone healing process. In addition, in vitro conditions used for testing the delivery kinetics of RNA therapeutics from biomaterials differ strongly from the complex, dynamic in vivo environment which is characterized by a highly orchestrated interplay of cells and mechanical and biochemical signals. Furthermore, various processing parameters of biomaterials are mutually dependent, which complicates optimization of these parameters considerably. Therefore, advanced design strategies such as Design of Experiments ​and computational modeling may help to capture the intrinsic complexity of these systems. In the future, biomaterial-based RNA delivery should be studied in 2D/3D models under dynamic conditions, while longitudinal in vivo monitoring of spatiotemporal delivery kinetics should provide insight into the effect of delivery kinetics of RNA complexes on in vivo bone healing responses. In addition, advanced technologies may allow to better mimic the temporal sequence of factors expressed during bone healing by making use of on-demand release systems and/or co-delivery of multiple biomolecules to create physiological feedback loops.

The article "Designing biomaterials for the delivery of RNA therapeutics to stimulate bone healing" was published in 2021. Journal: Mater Today Bio.

RNA therapy is still in its infancy with only few RNA-therapeutic approved for clinical use. To facilitate clinical translation, preclinical testing should provide proof-of-concepts in clinically relevant (animal) models and their alternatives. Importantly, regulatory compliant upscaling of sterilizable RNA-loaded biomaterials is required to enable clinical translation of RNA-delivering biomaterials with unsurpassed regenerative capacity.

## Funding

The authors would like to thank 10.13039/501100003246Netherlands Organization for Scientific Research (NWO, project 17615) for funding this research.

## Declaration of competing interest

The authors declare that they have no known competing financial interests or personal relationships that could have appeared to influence the work reported in this paper.
